The article "Effect of sex and rearing system on the quality and mineral content of fiber from raeini cashmere goats" was published in 2012. Journal: J Anim Sci Biotechnol.

# Effect of sex and rearing system on the quality and mineral content of fiber from raeini cashmere goats

**DOI:** 10.1186/2049-1891-3-20

**Published:** 2012-06-25

**Authors:** Mehrdad Shamsaddini-Bafti, Mahnaz Salehi, Ali Maghsoudi, Ali Mostafa Tehrani, Farhad Mirzaei, Syed Mojtaba Syed Momen

**Affiliations:** 1 Razi Vaccine & Serum Research Institute, Kerman Branch, 76175, Kerman, Iran; 2 Animal Science Research Institute of Iran, Dehghan Villa, 31585, Karaj, Iran; 3 Department of Agriculture, Faculty of Animal Science, Tarbiat Modares University, Tehran, Iran

**Keywords:** cashmere fiber, mineral contents, Raeini goat

## Abstract

The aim of this study was to compare the quality characteristics and mineral content of the fiber from male and female cashmere goats raised under different management systems. Male and female Raeini cashmere goats (<1.5 years of age, n = 48) were selected from flocks raised at a government breeding station or raised commercially under either rural or nomadic conditions. The staple length, cashmere fiber diameter, coefficient of variation for fiber diameter, percentage of cashmere in a fleece, percentage of guard hair in a fleece and cashmere tenacity averaged 4.6 ±0.1 cm, 18.0 ±0.1 μm*,* 20.9 ± 0.4%, 66.1 ± 1.5%, 33.8 ± 1.5% and 1.8 ± 0.2 gf/tex, respectively. The sulfur, copper and zinc content of the cashmere averaged 2.8 ± 0.1%, 0.00065 ± 0.00002% and 0.01276 ± 0.00025%, respectively. Rearing method significantly affected staple length, coefficient of variation of fiber diameter, cashmere tenacity and copper content. Males had a higher coefficient of variation of fiber diameter and cashmere tenacity than females (*P* < 0.05).

## Introduction

Despite the availability of inexpensive, flexible and stable synthetic fibers, the demand for cashmere is growing, presumably because of the revolutionized distribution of wealth around the world which has increased the demand for luxury items such as cashmere textiles [1]. The top quality cashmere (14 to 15 μm), which is used in knitted garments, comes from China (including inner and outer Mongolia) while the lower quality cashmere (17 to 18 μm) used in weaving comes mainly from Iran [2].

The down fiber content of commercial raw cashmere can vary between 15 and 90% depending on the coat type and the sorting method used in the country of origin. The ratio of inner coat (by weight) varies from 22 to 88% in Chinese, 20 to 60% in Indian, and 36 to 96% in Russian cashmere goats, as well as from 8 to 58% in Australian and 30 to 60% in Scottish semi-wild goats [3]. Iranian cashmere typically has an average down content of 74% ranging from a low of 56% to a high of 83% [4].

The goat population in Iran is estimated at 25.8 million head [5] and more than 5 million of these are pure cashmere goats. Pure cashmere goats are kept mostly in the eastern part of the country in the arid and semi arid zones surrounding the Loot desert. The Raeini goat is one of the most famous cashmere breeds raised in Iran [6]. It is raised in large numbers in the Kerman province of Iran where goat production contributes significantly to the agricultural economy. In this region, farmers keep goats for meat, milk and cashmere, but little effort is made to select and breed better quality cashmere goats. The mean weight of the fleece produced is 400 g ranging from 130 to 1,100 g per head. Down yield of raw cashmere fibers ranges between 30 and 70% and averages 16 to 19 μm in diameter and 4 to 7.5 cm in staple length [7].

Unlike mohair, cashmere quality appears to be intensively affected by non-genetic factors a feature most likely arising because of the seasonal growth of cashmere compared with continuous growth in mohair. This means that cashmere quantity and quality are influenced by a wide range of factors such as the climate of the rearing region, year or season, time of shearing, as well as the strain of goat and the selective breeding scheme used [8]. However, the extent to which these factors affect cashmere quality has not been quantified. Therefore, this study was conducted to determine the effects of sex of goat and three rearing systems on the quality traits and mineral content of cashmere obtained from Raeini goats.

## Materials and methods

### Animals and management

Data were collected from 24 male and 24 female (<1.5 years of age) Raeini goats. Three flocks of goats (n = 16) were used including an intensively reared breeding station flock, as well as extensively reared rural and nomadic flocks. The breeding station flock was housed at a governmental farm located near the city of Baft in Kerman Province located in southeastern Iran [6]. Station flocks are used to introduce goats selected for improved cashmere weight and quality to villagers and nomadic holders. Goats in the station flock were offered supplementary feed for one month in the summer and three months in the winter when the does kidded.. The rural flock was owned by small holders around Baft city (29.3° N, 65.60° E; mean annual rainfall of 320 to 400 mm and 23 °C) while the nomadic flock was owned by grazing goat holders migrating between mountainous (in summer), and flat (in winter) pastures in Kerman province (29.3° to 30.29° N, 52.44° to 57.07° E; mean annual rainfall of 180 to 400 mm and 23° to 27 °C).

### Samples and fiber measurements

Standard methods [9] were used to collect the fleece samples from the goats. A patch of approximately 10 cm^2^ of both hair and down fibers was sampled from the last rib on the right side of the experimental animals. The samples were placed in nylon bags and labeled. Fleece characteristics including the percentage of cashmere in a fleece, the percentage of hair in a fleece, staple length, cashmere fiber diameter and coefficient of variation of cashmere fiber diameter were measured. The staple length was determined by placing the staple against a ruler. Three or four staples were randomly chosen from each sample. Locks from each sample were individually washed with warm water (45 °C) and a non-ionic detergent, rinsed in warm water (40 to 50 °C), and then dipped in dichloromethane alcohol to remove any residual grease not previously removed in washing. Care was taken to avoid disturbing the staple formation of the fibers to minimize the loss of shorter fibers. Samples were then air-dried.

A small portion of the samples were separated as sub-samples for hand dehairing. The visual subjective test was used to separate the fine (cashmere) and coarse (hair) fibers, and their dry weights were determined. The down fiber diameter was determined using a projection microscope technique in accordance with ASTM D2130 [10]. Each sub-sample was compressed and its’ fibers were cut from base to mid-staple with a Hardy microtome [10]. Over one hundred fibers from each sample were measured. Mean fiber diameter, the standard deviation and the coefficient of variation were calculated for each sample. The fibers were combed out from the protruding end to remove loose fibers and foreign materials as well as to secure partial parallelization of the fibers. Then, the tuft was reversed and combing was repeated from the other end. The clamped tuft was placed in the grips of a tensile testing machine (Model 4001, Instron. Limited, High Wycombe, UK.) with a load cell of 100 kg. The clamps were pulled up at the rate of 25 cm/min. After recording the breaking load, the broken fibers were weighed and breaking tenacity was calculated using Eq1 [11].

Breaking tenacity (gf/tex(= (b/M) × 2.54 × 10^-5^ (E. 1)

Where b is bundle breaking load in gram force (gf), and M is bundle mass in grams (g).

The mineral content of the cashmere was determined by atomic absorption spectrophotometer in a manner described in many published papers [7].

### Statistical analysis

The data obtained were statistically analyzed using the general linear model (GLM) procedure of the SAS software package [12]. the statistical model was as follows

(1) $$\gamma_{\text{ijk}}=\mu +\alpha_{i}+\beta_{j}+{\left(\alpha \beta \right)}_{\text{ij}}+\epsilon_{\text{ijk}}$$

Where $\gamma_{\text{ijk}}$ is the individual record of the percentage of cashmere in a fleece, the percentage of guard hair in a fleece, staple length, cashmere fiber diameter, coefficient of variation of fiber diameter, cashmere tenacity or minerals (sulfur, copper and zinc),  is the population mean, $\alpha_{i}$ is the effect of the i^th^ sex, β_j_ is the effect of the j^th^ rearing method, (αβ)_ij_ is the interaction between sex and rearing method and ϵ${}_{\text{ijk}}$ is the residual effect. A Pearson correlation test was used to determine the significance of the correlation of fiber traits with the mineral content of the cashmere. All values are expressed as least square means ± SEM and a *P* < 0.05 was considered to be statistically significant.

## Result and discussion

### Fleece traits

The quality and commercial value of cashmere is often optimized from fleeces with high yield, long staple length, white color, small diameter and minimum contamination with guard hairs [13]. Each of these quality attributes affects the speed of processing processed yield as well as yarn and fabric quality [14]. Mean values, variances and ranges for the recorded traits are presented in Table [Table T1].

**Table 1 T1:** Cashmere quality and mineral content of Raeini goats

**Traits**	**Mean ± SE**	**CV**	**Min**	**Max**
Staple length, cm	4.6 ± 0.1	22.2	2.8	7.7
Cashmere mean fiber diameter, μm	18 ± 0.1	4.7	15.6	19.5
Coefficient of cashmere mean fiber diameter, %	20.9 ± 0.4	14.7	15.6	27.2
Cashmere, %	66.1 ± 1.5	16.3	42	91.2
Guard hair, %	33.8 ± 1.5	16.3	7.8	58.0
Cashmere tenacity, gf/tex	1.8 ± 0.2	70.9	0.5	5.6
Sulfur, %	2.8 ± 0.1	19.4	1.5	4.8
Copper, %	6.5 × 10^-6^ ± 0.2 × 10^-6^	25.6 × 10^-6^	3.5 × 10^-6^	10.9 × 10^-6^
Zinc,%	127.6 × 10^-6^ ± 2.5 × 10^-6^	13.6 × 10^-6^	91.7 × 10^-6^	167.5 × 10^-6^

Previous studies on Raeini cashmere goats [15] showed that the percentage of down weight varied between 59 and 75%, a result similar to that observed in our research. Miller [3] recorded that the percentage of undercoat in sorted and raw Iranian cashmere varied from 65.8 to 74.1% and 32% in Iranian common goats. The values obtained for cashmere percentage (66.1 ± 1.5%) in this study are not in agreement with previous reports of cashmere percentage observed in commercial cashmere flocks (58 ± 3.6%) [16], adult bucks (33 ± 6.8%) and does (45 ± 2.6%) in Australia [17].

Since the length of dehaired cashmere markedly affects its’ price, there is a common interest in producing cashmere with the greatest length to maximize the amount of cashmere obtained after the dehairing process. The length of down fibers differ and vary from 2.5 to 16.5 cm in most reports [3]. Fine fibers with a diameter less than 18 μm and a length more than 40 mm are commercially suitable for the knitting industry while diameters more than 17 to 18 μm and in some cases 24 μm and lengths shorter than 40 mm are used in worsted yarn systems [18]. Previous research [20] established properties of follicle producing fibers in Chinese goats and reported that fibers obtained from secondary follicles varied from 12 to 18 μm in diameter and from 4 to 10 cm in length while the diameter and length of guard hair fibers that were produced from primary follicles were 30 to 90 μm and 6 to 22 cm, respectively. The staple length of Raeini goats in this study was between 2.8 and 7.7 cm (Table 1).

The cashmere diameter in our study averaged 18 ± 0.12 μm (Table 1). A previous value for cashmere diameter published for this breed was 18.5 ± 0.1 μm [8], which supports our findings. However, other reported values of 19.5 to 20.2 μm [20], 19.3 μm [21] and range of 18.9 to 19.6 μm [20] for different flocks of Raeini cashmere goats are not completely in agreement with our findings. McGregor [22] reported the main sources of variation for cashmere produced from goats in the Pamir Mountain Districts of Murghab, Shugnon and Vanj in Tajikistan. In early spring 2010, for females, the means (sd) for mean fiber diameter, fiber curvature and staple length were 16.5 (1.7) μm; 46 (12.1) mm; 53 (22.9) mm respectively. Mean fiber diameter was affected by district, staple length and age of goat. Staple length was affected by district, mean fiber diameter, gender, age of goat and village. fiber curvature was affected by district, mean fiber diameter, shade of cashmere, age of goat and farmer. Cashmere from Vanj district was finer and shorter than cashmere from Murghab and Shugnon.

The “handle” of a textile product is generally referred to as softness and is a different property to prickle discomfort (more spinning fineness) and can be evaluated using easily obtained measurements of fiber diameter distribution. As shown in Table 1, the coefficient of variation for cashmere diameter was 20.9 ± 0.4%. Results of samples obtained from manufacturers in Europe, Iran, China, Australia and other countries have shown that the mean coefficient of variation of diameter from the dehaired cashmere samples was 22% with little variation around the median [23]. The coefficient of variation for cashmere diameter of Raeini cashmere goats was 16 to 22% which is in accordance with corresponding data (15.6 to 27.2%) obtained from other studies [14,24]. In contrast, this parameter in Sistan and Baluchestan native goat fleece was 19.6% ranging from 13 to 31% [24], and for Birjandi cashmere goats ranged from 19 to 31% [25].

The bundle strength of tops is rated as the third most important fiber property with respect to yarn strength and the speed of processing operations after mean fiber diameter and fiber length [26]. In the dehairing of cashmere, repeated mechanical action causes fiber breakage. Higher tenacity and more extensible fibers result in less fiber breakage and the potential use of the fiber in the worsted spinning system [22]. The results of our study demonstrated a value 1.76 ± 0.19 gf/tex for this trait and also indicated a large variation (70.9%) between samples in cashmere tenacity from 0.5 to 5.60 gf/tex (Table 1). This is different from other values for this breed (3.46 ± 0.5 gf/tex) observed [27].

### Mineral content

Sulfur is most important mineral utilized in the biosynthesis of methionine and cysteine which are essential components of all proteins. These sulfur-containing amino acids are effective in the activity of fiber producing follicles and thus stimulate fiber growth and improve fleece quality in the sheep or goat [28,29].

Both zinc and copper are indispensable micronutrients for fast growing tissues such as fiber-producing follicles [30]. Copper deficiency results in impaired keratinization of hair and wool and physical properties of wool like crimp that are dependent on disulfide groups. Thus, sheep exposed to sulfur deficiencies have shown lower sulfur content in their wool compared with a nutritionally adequate group [30,31].

The results of the present study show that the sulfur, copper and zinc contents of cashmere were in the range of 1.5 to 4.8%, 0.00035 to 0.00109% and 0.00917 to 0.01675%, respectively (Table 1). The copper content was significantly affected by rearing method (*P* < 0.05; Table 2). An average value of 4 ppm for copper in goat fiber has been reported [32].

**Table 2:** Effect of sex and rearing method on the mineral content of fiber from Raeini goats

**Effects**		**No.**	**Mineral (%)**		
			**Sulfur**	**Copper**	**Zinc**
Sex	Male	24	2.9 ±0.1	6.4 × 10^-6^ ± 0.33 × 10^-6^	126.0 × 10^-6^ ± 3.48 × 10^-6^
	Female	24	2.8 ± 0.1	6.6 × 10^-6^ ± 0.33 × 10^-6^	129.0 × 10^-6^ ± 3.48 × 10^-6^
*P* value			Ns	ns	ns
Rearing method	Breeding station	16	2.9 ± 0.1	7.1 × 10^-6^ ± 0.4 × 10^-6^	128.0 × 10^-6^ ± 4.3 × 10^-6^
	Rural	16	2.8 ± 0.1	5.7 × 10^-6^ ± 0.4 × 10^-6^	134.0 × 10^-6^ ± 4.3 × 10^-6^
	Nomadic	16	2.7 ± 0.1	6.7 × 10^-6^ ± 0.4 × 10^-6^	121.0 × 10^-6^ ± 4.3 × 10^-6^
*P* value			Ns	*	ns

^*^P < 0.05; ns: Not Significant.

Variable effects of dietary sulfur on zinc content in cashmere fiber of Raeini kids have been shown [30]. A decreased cashmere zinc content of 0.01165 to 0.01015% was reported with diets containing 0.22 or 0.14% sulfur [30]. In addition, a negative linear relationship between dietary sulfur and cashmere copper was reported so that at dietary levels of 0.4 and 0.14% sulfur, cashmere copper levels were 24.9 and 22.3 mg/kg, respectively [30]. The ranges of sulfur, copper and zinc in cashmere fibers of Raeini kids were 1.8 to 7%, 10 to 15 mg/kg and 75 to 299 mg/kg, respectively. The results of present study are in close agreement with previous results [20,33].

In fiber, sulfur was positively correlated with zinc content and negatively correlated with copper content. The correlation between zinc content and cashmere tenacity was high and negative (−0.24). There was a positive correlation between zinc and copper content in fiber (*P* < 0.05). However, the correlation between sulfur, copper and zinc with cashmere diameter (0.1,–0.7 and–0.04, respectively) was only significant between cashmere diameter and copper [33].

### Sex effect

The sex of goat did not significantly affect the mineral composition of cashmere fibers, although there were some differences between two sexes in the physical characteristics of their fleeces. The study showed that none of the measured parameters except for the coefficient of variation of cashmere fineness and cashmere tenacity (staple strength) was influenced by sex of goat (*P* <0.05; Table 3). Male fiber showed significantly stronger staple strength than female fiber (2.1 ± 0.2 and 1.4 ± 0.2 gf/tex; Table 3). This response is consistent with the slightly higher fiber sulfur content for males than females. Female goats tended to have more cashmere percentage and copper and zinc contents than males but these differences were not statistically significant (Table 2). In Australian cashmere goats, males tended to have a lower body weight and cashmere weight than females, but both sexes were similar in diameter and length of fibers [34]. Unlike Australian goats, in Chinese goats at all ages, males have coarser cashmere than females with an increasing trend as their age increased. Another research work reported that adult males were significantly heavier than adult females in cashmere weight, fiber diameter and length, and body weight [36]. It has been shown that an adjustment for sex and age effects would be necessary for fleece weight and fiber diameter for Angora goats in Argentina [36].

**Table 3:** Effect of sex and rearing method on staple length (SL), cashmere percentage (C), cashmere mean fiber diameter (CFD), coefficient of cashmere diameter (CVFD) and cashmere tenacity (CT) of Raeini goats

**Effects**		**No.**	**Traits**				
			**Sl, cm**	**C, %**	**VFD, μm**	**CVFD, %**	**CT, gf/tex**
Sex	Male	24	4.8 ± 0.2	64.1 ± 2.1	18.0 ± 0.2	21.7 ± 0.6	2.1 ± 0.2
	Female	24	4.4 ± 0.2	68.2 ± 2.1	18.0 ± 0.2	20.0 ± 0.6	1.4 ± 0.2
*P* value			ns	ns	ns	*	*
Rearing method	Breeding station	16	4.8 ± 0.2	70.1 ± 2.6	17.9 ± 0.2	21.5 ± 0.7	2.6 ± 0.3
	Rural	16	4.0 ± 0.2	64.2 ± 2.6	18.1 ± 0.2	19.3 ± 0.7	1.3 ± 0.3
	Nomadic	16	5.0 ± 0.2	64.2 ± 2.6	17.9 ± 0.2	21.8 ± 0.7	1.3 ±0.3
*P* value			*	ns	ns	*	**
Sex × Rearing method *P* value			ns	ns	**	ns	ns

^*^P < 0.05; ^**^P < 0.001; ns: Not Significant.

Results obtained from black and brown goats from Birjand in eastern Iran showed that the means of 3,250 records for fleece weight and down fiber percentage, length and diameter of cashmere fibers in raw fleece were 319.4 ± 125.7 g, 148.5 ± 58.3 g, 47.5 ± 8.9 mm and 16.6 ± 1.2 μm, respectively. In these goats, the effects of flock, region, sex and type of birth were significant for these parameters [25].

A previous study indicated that the effect of sex was significant on cashmere percentage, fiber diameter and staple length of Raeini goats and the amount of cashmere fibers for males and females was 63 ± 10% and 68 ± 10%, fiber diameter was 21 ± 2.1 and 19.4 ± 1.7 μm; and length of fiber was 6.4 ± 1.9 and 6.5 ± 1.8 cm, respectively [9]. Another study reported that the staple strength of cashmere fibers in two-year old males (mean body weight 24.9 ± 2.5 kg) was between 3.2 and 3.7 gf/tex [37]. No significant difference has been observed between male and female goats in down fiber strength (0.3 ± 0.1 versus 0.4 ± 0.1 gf/tex) [38].

### Rearing method

Staple length was significantly different between rural goats, nomadic goats and goats kept at a breeding station. Also, there was an interaction between sex and flock for cashmere fiber diameter (*P* < 0.001; Table 3). Coefficient of variation of cashmere fineness, cashmere tenacity and cashmere copper was also influenced by the rearing method (Tables 3 and 2).

More fleece weight, staple length and down fiber percentage was observed in goats reared in station flocks compared with a rural system [33]. A large variation in both cashmere production and length, as well as on the percentage of active follicles among different temperature/humidity locations was found [37], although fiber diameter and cashmere growth rate were not affected. There were effects of cashmere origin and processor on the properties of dehaired cashmere [23,39]. It has been reported that the main sources of variation for staple length and fiber diameter in Pamir mountain cashmere goats were district and age of goat [18]. Other researchers observed that the sulfur, copper and zinc content in cashmere fibers of rural flocks were lower than the goats of breeding station flocks. They demonstrated that the sulfur content of cashmere for station (3.2 ± 0.4%) and rural (2.9 ± 0.5%) goats was significantly different, but there were not significant differences in copper and zinc content of cashmere fibers for station (0.00122 ± 0.00011% and 0.00119 ± 0.00014%) and rural (0.02048 ± 0.00355% and 0.02017 ± 0.00350%) flocks [33].

## Conclusions

In this study, the fiber diameter of dehaired cashmere samples ranged from 15.59 to 19.51 μm. The cashmere yield ranged from 42 to 91.2% and there was a high distinction in cashmere tenacity. The sulfur, copper and zinc contents of cashmere were in the range of 1.5 to 4.8%, 0.00035 to 0.00109% and 0.00917 to 0.01675%. There was a slight correlation between cashmere mineral content and quality. Therefore, these parameters may be good variables for selecting and improving goats to produce better quality cashmere. There are cashmere goats in the Murghab, Shugnon and Vanj districts of Tajikistan which produce the high quality cashmere, comparable to the premium grades of Chinese cashmere. There is substantial scope to increase the commercial value of cashmere produced by goats in Tajikistan, in particular by increasing staple length for fine cashmere, reducing mean fiber diameter for the longest cashmere and ensuring cashmere has an acceptable fiber curvature and a white color.

## Competing interest

The authors declare that they have no competing interests.

## Authors’ contribution

Mehrdad Shamsaddini Bafti conceived of the study, and carried out the animal trail, finished the statistical analysis and drafted the manuscript. Mahnaz Salehi, Ali Maghsoudi, Ali Mostafa Tehrani and Syed Mojtaba Syed Momen participated in sampling, Lab works and related studies. Farhad Mirzaei was editor and designer of final report. All authors read and approved the final manuscript.
